# Screening of Biomarkers in Liver Tissue after Bariatric Surgery Based on WGCNA and SVM-RFE Algorithms

**DOI:** 10.1155/2023/2970429

**Published:** 2023-01-30

**Authors:** Yicheng Jiang, Yu Wang, Shuai Chen, Zhixin Liu, Haojun Yang, Yuwen Jiao, Liming Tang

**Affiliations:** Center of Gastrointestinal Disease, The Affiliated Changzhou No. 2 People's Hospital of Nanjing Medical University, Changzhou, China

## Abstract

As the most common chronic liver disease around the world, nonalcoholic fatty liver disease (NAFLD) has a close connection with obesity, diabetes, and metabolic syndrome. Bariatric surgery (BS) is considered to be the most effective treatment for NAFLD. However, the regulatory mechanism of hepatic lipid metabolism after BS remains poorly elucidated. By analyzing two transcriptome datasets regarding liver tissues after BS, namely, GSE83452 and GSE106737, we acquired 110 differentially expressed genes (DEGs). By further analysis of DEGs in terms of the weighted gene coexpression network analysis (WGCNA) and support vector machine-recursive feature elimination (SVM-RFE) algorithms, we identified four crucial genes participating in the regulation of hepatic lipid metabolism: SRGN, THEMIS2, SGK1, and FPR3. In addition, the results of gene set enrichment analysis (GSEA) showed that BS can activate immune-related regulatory pathways and change immune cell infiltration levels. Finally, through cellular level studies, we found that the silencing of SRGN affects the expression of SREBP-1, SIRT1, and FAS during adipogenesis in the liver and the formation of lipid droplets in the liver. In summary, the immune system in the liver is activated after BS, and SRGN participates in the regulation of hepatic lipid metabolism.

## 1. Introduction

Nonalcoholic fatty liver disease (NAFLD), as the most common chronic liver disease, influences approximately a quarter of the global population [1]. NAFLD contains a series of pathological changes, including nonalcoholic fatty liver (NAFL) and nonalcoholic steatohepatitis (NASH). Pathological features of NAFL are the presence of macrovesicular steatosis in >5% of hepatocytes, meanwhile excluding liver damage caused by excessive alcohol consumption. NASH is characterized by the presence of hepatic steatosis and inflammatory damage to hepatocytes (enlargement of hepatocyte balloons), with or without fibrosis [2].

In addition to causing chronic liver diseases such as hepatocellular carcinoma and liver cirrhosis, NAFLD is closely related to a variety of systemic metabolic diseases, including hypertension, obesity/overweight, and type 2 diabetes [3, 4]. Some experts have proposed that the disease can be more accurately described as metabolic-associated fatty liver disease (MAFLD) to better reflect pathogenesis and heterogeneity of patients. Diagnostic criteria for MAFLD should be based on evidence of liver steatosis such as liver biopsy histology, blood biomarker testing, or imaging, with at least one of these conditions: overweight/obesity, metabolic dysfunction, and type 2 diabetes [5].

Currently, NAFLD has no approved drug treatments, and the main treatment is diet control and increased exercise. However, it is difficult to improve NAFLD through lifestyle interventions. Studies have found that the degree of weight loss is closely and positively correlated with the improvement of steatosis. Only weight loss of ≥3% can relieve steatosis, and ≥5% weight loss can improve inflammation while fibrosis can be reduced by ≥10% weight loss [6, 7]. Against this background, more and more pharmacological interventions for NAFLD are proposed. These investigational drugs target the following aspects: metabolic disruption, inflammatory responses, oxidative stress, inflammatory signaling, apoptosis, and fibrosis [8]. In addition, there is evidence that gut microbiota has an impact on liver function, contributing to obesity and NAFLD [9, 10]. Recent studies have found that fecal microbiota transplantation (FMT) improves insulin resistance, proinflammatory cytokines, and intrahepatic lipid accumulation in mice [11, 12]. Nevertheless, since the fact that reducing excess visceral fat is a key approach to improve hepatic steatosis, bariatric surgery plays a key role in the treatment of NAFLD by reducing abdominal obesity [13].

According to the latest guidelines [14], patients with NAFLD can undergo BS when lifestyle modifications and drug interventions are ineffective. BS has now proven to be the most effective method to maintain long-term weight loss, which both benefits NAFLD and reduces mortality from other related chronic diseases such as diabetes, heart disease, and cancer, especially in elderly patients [15–17]. Mummadi et al. reported significant improvements in liver steatosis, steatohepatitis, and fibrosis after BS with liver biopsy results [18]. In addition, biochemical indicators such as ALT, AST, ALP, and GGT were found to be significantly reduced after BS [19]. Interestingly, a meta-analysis of treatments for weight loss showed that BS showed a weaker dose-response relationship between weight loss and the degree of liver prognosis compared to other types of treatments [20].

The mechanism of NAFLD progression is usually explained with the classic “multiple hit” theory, which states that as a result of cumulative triglyceride accumulation, endoplasmic reticulum stress response, protein misfolding, oxidative stress, and mitochondrial damage are produced by cell stress, causing a prolonged state of chronic inflammation and resulting in the hyperactivation of immunity and inflammation in liver tissue [21]. It has been found that liver inflammation and liver damage can be triggered and amplified by innate and adaptive immune activation, which contributes to NAFLD/NASH, and the activation of immune system can recruit dendritic cells, neutrophils, and CD8+ T cells [22–25]. However, the potential mechanism by which BS improves NAFLD remains to be explored.

Bioinformatic analysis techniques are widely applied to find potential biomarkers and patterns. Zhang et al. acquired the differential genes in liver tissue after BS from the GEO database and obtained LCP1, a key gene that regulates liver inflammation through WGCNA and PPI networks [21]. Chen et al. analyzed the data on BS influencing the subcutaneous adipose tissue transcriptome expression in GEO databases and obtained key genes that regulate fat differentiation through WGCNA, SVM-RFE algorithms, and LASSO logistic regression and verified them [26].

Our study analyzed transcriptome data in liver tissue after BS surgery and obtained 110 DEGs. The key genes regulating liver lipid metabolism were obtained by WGCNA and SVM-RFE algorithms, their correlation with immune cells was analyzed by GSEA, and the regulatory effect of crucial genes in liver lipid metabolism was further verified.

## 2. Materials and Methods

### 2.1. Data Collection and Processing

Two microarray datasets regarding liver tissues after BS were retrieved in the GEO database (Table 1). GSE83452 and GSE106737 were merged via the R packets in SilicoMerging [26], and then, the empirical Bayesian methods were used to adjust the batch effects. By using the limma V3.42.0 packets with a standard of |log(fold change, FC)| > 1.5, DEGs in postoperative liver tissue samples were figured out. Volcano maps and Venn maps were created using Sangerbox 3.0, which preserved overlapping DEGs for further analysis.

### 2.2. Functional Correlation Analysis

To analyze overlapping DEGs, we applied the “clusterProfiler” and the “http://org.Hs.eg.db” R package for Gene Ontology (GO) annotations and the Kyoto Encyclopedia of Genes and Genomes rest API for KEGG gene annotations. The above results are displayed in the form of a circle chart and a column chart (http://soft.sangerbox.com/).

### 2.3. Screening and Verification of Biomarkers

We utilized support vector machine-recursive feature elimination (SVM-RFE) and weighted gene coexpression network analysis (WGCNA) to figure out biomarkers for NAFLD. First, we performed the WGCNA package in R software to construct a coexpression network for the modules most relevant to the phenotype. The network was established after handling missing values and outliers. The key module was screened by correlation analysis, and the genes with the strongest correlation with BS were identified based on the key modules. Then, the “e1071” R package was performed to further analyze DEGs by SVM-RFE. Finally, the results of the above analyses were intersected.

### 2.4. Gene Set Enrichment Analysis

The GSEA software and the subset “c2.cp.kegg.v7.4.symbols.gmt” were downloaded from the GSEA website and the Molecular Signatures Database, respectively. We divided all samples into pre-BS and post-BS groups and then analyzed the potential pathways and molecular mechanisms by GSEA, with one thousand random combinations. Statistical significance was set at *P* < 0.05 and FDR < 0.25.

### 2.5. Cell-Type Enrichment Analysis

The CIBERSORT was performed in RStudio to analyze the proportion of 22 types of immune cells in the liver. The original enrichment score and immune score were obtained by using the gene expression profile data. To explore the relationship between biomarkers and the proportion of immune cell infiltration, we used Spearman's rank correlation analysis in R software. The “ggplot2” package was utilized to visualize the results.

### 2.6. Hepatocyte Culture and Induction

We obtained the hepatoma carcinoma cell line (HepG2 cells) from the National Biological Cell Culture Center (Shanghai, China), as a model of hepatocyte metabolism and biosynthesis. Under constant temperature and humidity (37°C, 5% CO_2_), HepG2 cells were cultured in Dulbecco's Modified Eagle's Medium (DMEM) (Gibco, China) containing 10% fetal bovine serum (FBS) (Gibco, China) and 1% penicillin/streptomycin. Using a normal medium as a control, model group cells were incubated with 500 *μ*M FFA (oleic acid and palmitic acid, 2 : 1) in DMEM containing 10% fat-free bovine serum albumin (BSA) to stimulate lipid accumulation for 24 h [27].

### 2.7. Oil Red O Stain

The first step is to dissolve Oil Red O powder (Sigma) in isopropanol, followed by dilution 3 : 2 with distilled water. Then, we fix the cells with 4% polymethanol for 30 min. A microscope was used to observe and photograph the stained cells after washing them three times with PBS and staining them with Oil Red O for 30 min [26].

### 2.8. Quantitative PCR Analysis

The RNA was extracted from samples using TRIzol, and Vazyme HiScript II Q RT SuperMix (Vazyme, China) was used for reverse transcription. The RT-PCR reactions were carried out as follows: 5 min at 37°C, 5 sec at 85°C, and final reduction to 4°C. qPCR was carried out using SYBR Premix Ex Taq II (Vazyme, China). The primers used (Sangon Biotech, China) are listed in Table 2. The GAPDH was utilized as an internal reference to calculate the relative mRNA expression of target genes by the 2^−(*ΔΔ*Ct)^ method.

### 2.9. Western Blotting

We used a radioimmunoprecipitation assay (RIPA) buffer containing 1 mM phenylmethylsulfonyl fluoride (PMSF) (Beyotime, China) to extract the total protein. Total protein was added to SDS-PAGE at 8%, blotted onto nitrocellulose membranes, and then blocked with a blocking buffer (Beyotime, China) for 2 hours. The membranes were incubated with primary antibody SREBP-1c, FAS, SIRT1, and *β*-actin for 1 hour at room temperature or overnight at 4°C. We obtained the primary antibodies from AiFang. After being washed 3 times in TBST, the blot was then incubated with horseradish peroxidase-conjugated secondary antibodies (Beyotime, China) for 1 hour. The ECL chemiluminescence kit (Thermo Scientific, USA) was used to detect immunoreactive bands.

### 2.10. Cell Transfection

SRGN gene-specific si-RNA was obtained from Ribio. We first inoculated cells in 6-well plates and transfected si-RNA (concentration 50 nmol) when cell confluency reached 60%-80%. After 24 h of transfection, HepG2 cells were inducted by FFA for 24 hours.

### 2.11. Immunofluorescence Analysis

After antibody incubation according to instructions, the expression levels of immunofluorescence-labeled SREBP-1c/FAS/SIRT1 were detected with an fluorescent inverted microscope (IX71-DP73, Olympus Microsystems).

### 2.12. Statistical Analysis

All statistical analyses were carried out using SPSS 22.0 (SPSS statistics, USA). The GraphPad Prism 7.0 (GraphPad Software, USA) was used to generate charts and plots. Student's *t*-test was utilized to compare statistical differences.

## 3. Results

### 3.1. DEG Screening after BS

First, we merged the two datasets GSE83452 and GSE106737. Afterwards, we eliminated batch effects so that the distribution of data between the two datasets would be unanimous (Figures 1(a) and 1(b)) and the samples clustered together (Figure 1(c)). Then, we set |logFC| > 1.5 and *P* < 0.05 as defined criteria and then screened 110 DEGs from GSE83452 and GSE106737, including 26 upregulated DEGs and 84 downregulated DEGs (Figures 1(d) and 1(e) and Table 3).

### 3.2. GO and KEGG Pathway Enrichment Analyses

We performed GO annotation and KEGG analysis for further enrichment analysis of DEGs. For the biological process (BP), DEGs were mainly enriched in response to inorganic substance, abiotic stimulus, oxygen-containing compound, metal ion, and cellar response to inorganic substance (Figure 1(f)). For the cellular component (CC), DEGs were mainly enriched in the perinuclear region of the cytoplasm, transcription factor AP-1 complex, mitochondria-associated ER membrane, organelle membrane contact site, and M band (Figure 1(g)). Regarding the molecular function (MF), 14-3-3 protein binding, vasopressin receptor binding, protein tyrosine/threonine phosphatase activity, ammonia-lyase activity, and insulin-like growth factor II binding were significantly enriched (Figure 1(h)). In addition, the enriched KEGG mainly includes 8 pathways: mineral absorption, IL-17 signaling pathway, TNF signaling pathway, osteoclast differentiation, viral protein interaction with cytokine and cytokine receptor, Toll-like receptor signaling pathway, NOD-like receptor signaling pathway, and chemokine signaling pathway (Figure 1(i)).

### 3.3. Construction of WGCNA and Module Identification of NAFLD after BS

After filtering out the missing values, we formed a sample cluster tree with the remaining 74 samples and 7875 genes (Figure 2(a)). We set the power of *β* = 7 as the soft thresholding parameter to ensure a scale-free network (Figure 2(b)). The WGCNA package was executed in RStudio to construct a coexpression network, including 17 modules (Figure 2(c)). It turned out that the green-yellow module has the strongest correlation between the pre-BS and post-BS groups, with 59 genes involved (Figure 2(d)). In addition, we further analyzed the importance of DEGs in the green-yellow module after BS (Figure 2(e)).

### 3.4. Identification of Optimal Biomarker

The SVM-RFE algorithm was used to further screen DEGs to obtain 4 important key genes (Figure 3(a)). By intersecting the analysis results of SVM-RFE and WGCNA, we obtain four important indicators: SRGN, THEMIS2, SGK1, and FPR3 (Figure 3(b)). The expression of SRGN, THEMIS2, SGK1, and FPR3 was significantly different in the combined dataset (Figure 3(c)). Results showed that the expression levels of SRGN, THEMIS2, SGK1, and FPR3 decrease significantly in liver tissue after BS, which is an important regulatory gene for NAFLD after BS.

### 3.5. Gene Set Enrichment Analysis and Immune Cell Infiltration Results

We further evaluated the relevant pathways and molecular mechanisms via GSEA and found that the B cell receptor signaling pathway, T cell receptor signaling pathway, NOD-like receptor signaling pathway, leukocyte transendothelial migration, and natural killer cell-mediated cytotoxicity were activated after BS (Figure 4(a)). It turned out that the changes in the proportion of immune cell infiltration after BS were mainly concentrated in B cell naive, plasma cells, T cell CD4 naive, T cell CD4 memory resting, NK cell resting, mast cell resting, and neutrophils in the postoperative period (Figure 4(b)). The relative proportions of immune cells in the GSE83452 and GSE106737 datasets were further visualized with cumulative histograms (Figure 4(c)).

The expression of SRGN had a significant and positive connection with the degree of neutrophil, plasma cell, and T cell CD4 memory resting infiltration but a negative relation with the degree of mast cell resting and macrophage M0 infiltration (Figure 4(d)). The expression of THEMIS2 had a significant and positive connection with the degree of plasma cell, neutrophil, and NK cell-activated infiltration (Figure 4(e)). The expression of SGK1 had a significant and positive relation with the degree of neutrophil, plasma cell, and T cell CD4 memory resting infiltration while a negative connection with the degree of mast cell resting infiltration (Figure 4(f)). The expression of FPR3 had a close and positive connection with the degree of neutrophil, plasma cell, and T cell CD4 memory resting infiltration while a negative connection with the degree of NK cell resting, T cell CD8, and macrophage M0 infiltration (Figure 4(g)).

### 3.6. Silencing SRGN Expression Inhibits Lipid Accumulation in HepG2 Cells

First, the ability of FFA to induce HepG2 cell adipogenesis was verified by staining Oil Red O on the HepG2 cell. The results showed that adding FFA to HepG2 cells can promote lipid accumulation (Figure 5(a)). After 24 hours of FFA induction, the expression level of SRGN was significantly increased. In addition, the expression levels of SREBP-1 and FASN were also remarkably increased after stimulation with FFA for 24 hours while the expression levels of SIRT1 were decreased (Figure 5(b)). Then, we verified the silencing efficiency of si-RNA and found that si-SRGN#2 and si-SRGN#3 have higher silencing efficiency (Figure 5(c)). The effect of silencing SRGN on HepG2 was observed 24 hours after FFA induction. We found that the silencing of SRGN influenced the expression levels of SREBP-1, SIRT1, and FASN proteins (Figures 5(d) and 5(e)) and reduced the formation of the lipid droplet (Figure 5(f)). The results demonstrated that SRGN contributed to regulating hepatic lipid metabolism.

## 4. Discussion

Currently, NAFLD is considered to be the most common chronic liver disease [1] and is closely related to the metabolic syndrome, involving various pathogeneses, connected with a multitude of uncertain risk factors such as lifestyle, metabolic, genetic, and microbial-related factors [21]. The development of NAFLD includes several stages. First, the accumulation of lipids in hepatocytes leads to simple steatosis. Then, as inflammatory injuries worsen, the disease progresses to NASH, with or without fibrosis. If fibrosis continues to grow, the disease ends in cirrhosis and even hepatocellular carcinoma [28]. There is evidence that BS can significantly improve metabolic dysfunction, reduce lipid accumulation, and help to alleviate the progression of NAFLD/NASH [29]. However, the potential mechanism by which BS relieves NAFLD/NASH still needs to be further investigated. By conducting related bioinformatic analysis of the preoperative and postoperative gene expression data of liver tissues in patients with NAFLD, the potential mechanism of bariatric surgery to improve hepatic lipid metabolism and reduce lipid droplet formation in the liver was further revealed, which provided new insights for the research and clinical treatment of NAFLD.

Through bioinformatic analyses based on GEO datasets of GSE83452 and GSE106737, we could discover the changes in gene expression levels in liver tissues after BS which can reveal underlying pathways of hepatic steatosis and inflammation relief. We identified a total of 110 DEGs, including 84 upregulated DEGs and 26 downregulated DEGs.

The enrichment analysis was performed to evaluate the main role of overlapping DEGs. For the biological process (BP), DEGs were mainly enriched in response to an inorganic substance, to an abiotic stimulus, and to an oxygen-containing compound. Previous studies suggested that hepatocyte injury in NASH encompasses a variety of features, such as endoplasmic reticulum (ER) stress [30], dysfunctional unfolded protein responses [31], inflammasome activation, inflammation and enhanced wound responses [32], and activation of apoptotic pathways [33].

The cellular component (CC) analysis showed that DEGs are mainly located in the perinuclear region of the cytoplasm, transcription factor AP-1 complex, mitochondria-associated ER membrane, organelle membrane contact site, and M band. The AP-1 complex can greatly affect cell proliferation and neuronal activation, while participating in apoptosis induced by cell stress, DNA damage agents, or lack of survival signals [34]. In addition, mitochondria-associated endoplasmic reticulum (ER) membranes play a vital role in detecting hepatocyte nutrient status and energy metabolism, especially in the exchange of substances such as Ca^2+^ and ROS, which are required for metabolic homeostasis. First, disturbance of Ca^2+^ homeostasis induces UPR within the ER, followed by the production of ROS and the entry of ROS into the mitochondria. Along with ROS, oxidative stress induction results in hepatic fat accumulation, steatosis, and progression of NAFLD by inducing hepatic IR, apoptosis, inflammation, and mitochondrial dysfunction [35, 36].

For the molecular function (MF), 14-3-3 protein binding, vasopressin receptor, protein tyrosine/threonine phosphatase activity, ammonia-lyase activity, and insulin-like growth factor II were significantly enriched. Out of the seven 14-3-3 isoforms, 14-3-3*ζ* is a member of an abundant family of scaffolding and chaperone proteins expressed in all eukaryotic cells and plays a vital role in visceral adipogenesis. Deficiency of 14-3-3*ζ* leads to aberrant expression of the hedgehog signaling factor Gli3 and the cyclin-dependent kinase inhibitor p27Kip1, thereby attenuating fat formation [37, 38]. In addition, the vasopressin receptor participates in the regulatory process of lipid metabolism in hepatocytes, which can promote glycogenation and gluconeogenesis in hepatocytes [39]. Furthermore, it has been reported that insulin-like growth factor II acts in response to the growth hormone (GH), thereby affecting hepatocyte differentiation, proliferation, and apoptosis [40].

By using CIBERSORT to analyze immune cell infiltration, we found a significant decrease in plasma cells, T cell CD4 memory resting, and neutrophils after BS. KEGG analysis demonstrated that five immune system-related pathways, the IL-17 signaling pathway, TNF signaling pathway, Toll-like receptor signaling pathway, NOD-like receptor signaling pathway, and chemokine signaling pathway, were significantly enriched. GSEA further confirmed the changes in the immune system of liver tissue after BS and found that multiple immune system-related pathways were activated after BS. It turned out that the B cell receptor signaling pathway, T cell receptor signaling pathway, NOD-like receptor signaling pathway, and natural killer cell-mediated cytotoxicity contributed to the occurrence and development of NAFLD/NASH and were involved in the inflammatory response and fibrosis of the liver [41–44]. There is increasing evidence that innate and adaptive immunities are driving forces in the process of liver inflammation and fibrosis [22, 45]. The results are largely connected with previous studies, which reveal the significant role of immune cell regulation in NAFLD/NASH.

The sirtuin family consists of seven family members (SIRT 1-7) with NAD-dependent deacetylases, deacetylases, and/or ADP-ribosyl transferases activities [46]. The NAD-dependent protein deacetylase sirtuin-1 (Sirt1) plays an important role in regulating glycolipid homeostasis and cell differentiation [47, 48]. Sirt1 was found to be involved in the regulation of NAFLD through a variety of molecular mechanisms. Ponugoti et al. found that Sirt1 deacetylates and inhibits the sterol response element-binding protein 1c (SREBP-1c) activation in the regulation of NAFLD [49]. Zhu et al. found that the combination of luteolin and lycopene can effectively improve NAFLD by activating the Sirt1/AMPK pathway [50]. Sirt1 was also found to activate the Wnt/*β*-catenin pathway, thereby promoting the recovery of liver fatty injury [51]. Another member of the sirtuin family, sirtuin 4 (Sirt4), is an ADP-ribosyl transferase that is expressed differently in the liver and is involved in regulating glucose/lipid homeostasis [52]. Previous studies found that downregulation of Sirt4 leads to increased oxidation of free fatty acids in the liver and muscles and that Sirt4 participated in the regulation of glucose metabolism by reducing amino acid-stimulated insulin secretion [53, 54]. Furthermore, Guo et al. found that Sirt4 could deacetylate and destabilize mitochondrial trifunctional protein *α*-subunit (MTP*α*), which inhibits lipid accumulation in hepatocytes [55]. In this paper, we focus on the Sirt1/SREBP-1c pathway, and further research on Sirt4 needs to be developed.

Thymocyte-expressed molecule involved in selection 2 (THEMIS2) is enriched in B cells and macrophages, functioning as a signaling scaffold to regulate Toll-like receptor (TLR) responses [56]. Through participation in pathogen-associated molecular patterns (PAMPs), TLRs promote the production of inflammation-related factors and mediators such as IL-6, TNF, and cyclooxygenase 2 (Cox2), which are involved in both the acute response to infection or trauma and pathogen-specific adaptive immune responses [57]. Our study shows that the expression of THEMIS2 has a significant and positive connection with the degree of plasma cell-, neutrophil-, and NK cell-activated infiltration, which may explain how THEMIS2 is involved in the immune pathway of liver inflammation. In addition, studies have found that lncRNA THEMIS2-211 is highly expressed in hepatocellular carcinoma (HCC) and has a connection with the poor prognosis of HCC patients [58]. They found that lncRNA THEMIS2-211 interacts with miR-940 and functions physiologically as an oncogene. HCC has been considered as a terminal stage of NAFLD. Whether THEMIS2 contributes to the progression of NAFLD into HCC remains to be further explored.

Serum glucocorticoid-regulated kinase 1 (SGK1) is a transcriptional target of steroid hormones, including aldosterone, glucocorticoids, and other stimuli such as glucose. SGK1 is activated by phosphoinositide 3-kinase and is located downstream of insulin signaling. Former studies have found that SGK1 participates in many physiological and pathophysiological processes and that excessive activation of SGK1 promotes inflammation and fibrosis [59]. Pietro et al. found that SGK1 was expressed in adipose tissue and influences adipocyte differentiation by regulating Foxo1 phosphorylation [60]. Li et al. further demonstrated that aldosterone and glucocorticoid stimulated the expression of SGK1 in differentiated 3T3-L1 adipocytes and that SGK1 was highly expressed in the adipose tissue of obese and type 2 diabetic mice and humans [61]. In addition, studies have confirmed that SGK1 is also expressed in the liver and is able to regulate insulin sensitivity [62]. Sierra-Ramos et al. found that the content of triglycerides in the liver tissue of SGK1-overexpressing mice was significantly increased and that the liver steatosis was more severe than that of ordinary mice via Oil Red O staining [63]. Whether SGK1 can affect liver adipogenesis and inflammatory responses through the immune system remains to be further investigated.

N-Formyl peptide receptor 3 (FPR3) is a G protein-coupled receptor involved in the recruitment and activation of immune cells [64]. FPR3 has been found in eosinophils, monocytes, macrophages, and dendritic cells [65]. Several FPR3 ligands have been identified, including F2L, an acetylated N-terminal fragment of human heme-binding protein [66], and the neuroprotective peptide humanin [67]. FPR3 participates in the regulation of anti-inflammatory processes in neutrophils [68]. In addition, Lee et al. found that FPR3 might regulate immune responses by regulating CD4 T cell activity [69]. However, no studies have linked FPR3 to liver adipogenesis and inflammatory responses. According to our study, the decrease of FPR3 expression in liver tissue after BS may be related to the changes of immune cells, which remains to be further studied.

SRGN is an intracellular proteoglycan mainly located in secretory vesicles [70, 71] and a major proteoglycan in inflammatory cells of white adipose tissue, including macrophages, T cells, mast cells, and platelets [72]. Studies have shown that SRGN is expressed in adipocytes and is induced to express during adipocyte differentiation [73]. In addition, further studies by Doncheva et al. found that SRGN was mainly expressed by immune cells in white adipose tissue and involved in the inflammatory process in white adipose tissue [74]. Furthermore, it has been found that SRGN expression correlates with plasma LDL levels [75] while acute and chronic inflammation frequently brings about changes in plasma LDL levels [76]. Our study showed that the expression level of SRGN tended to decrease in liver tissue after BS, while the silencing of SRGN could affect the expression of hepatic lipid metabolism pathway markers and affect lipid droplet formation. The results of our study might help to reveal the potential pathway and molecular mechanisms by which BS affects hepatic lipid metabolism and adipogenicity.

There are several limitations and shortcomings in our research. First, the data for this study were derived from public databases, with incomplete clinical information and a lack of external validation. Another limitation of our study is the choice of statistical methods used for data analysis and the accuracy of the database, which may influence the interpretation of the results. Finally, the sample size included in the analysis was relatively small and had regional and ethnic limitations.

## 5. Conclusion

In conclusion, we identified 110 genes whose expression was altered in liver tissue after BS. Furthermore, four key biomarkers, THEMIS2, SGK1, FPR3, and SRGN, were screened by WGCNA and SVM-RFE algorithms. In addition, it turned out that BS can activate immune regulatory pathways while neutrophils and plasma cells were significantly downregulated, and THEMIS2, SGK1, FPR3, and SRGN were significantly associated with immune cell infiltration. Finally, cell experiments confirmed that SRGN contributed to regulating hepatic lipid metabolism.

## Figures and Tables

**Figure 1:** DEG screening and analysis. (a–c) The merging of datasets was conducted by eliminating the batch effect so that the distribution of data had a tendency to be consistent, and the samples clustered together. (d) Heat map of 110 DEGs in the combined data. (e) Volcano plots of DEGs: red triangles represent 84 downregulated DEGs, and green circles represent 26 upregulated DEGs. (f–h) Gene Ontology (GO) enrichment analysis of all DEGs in terms of molecular function (MF), biological processes (BP), and cell composition (CC). (i) Kyoto Encyclopedia of Genes and Genomes analysis of all DEGs.

**Figure 2:** WGCNA analysis. (a) Construction of a sample cluster tree. (b) Calculating soft-thresholding power. (c) Cluster dendrogram after dynamic tree cut and dynamic merging. (d) Heat map of module-trait relationships depicting correlations between module eigengenes and bariatric surgery. (e) The gene significance for bariatric surgery in the green-yellow module. WGCNA: weighted gene coexpression network analysis.

**Figure 3:** Identification of relevant biomarkers after bariatric surgery. (a) Support vector machine-recursive feature elimination (SVM-RFE) identified 4 genes with the minimum RMSE. (b) Overlapping DEGs in SVM-RFE and the green-yellow module. (c) The expression of genes including SRGN, THEMIS2, SGK1, and FPR3 significantly downregulated after bariatric surgery in the merged data. ^∗^*P* < 0.05 and ^∗∗^*P* < 0.01. RMSE: root mean square error.

**Figure 4:** Immune infiltration of liver tissue and correlation between DEGs and infiltrating immune cells. (a) Pathway analysis using GSEA about bariatric surgery. (b) Analysis of liver immune cell infiltration after bariatric surgery. (c) Relative infiltrating proportion of immune cells in each sample. (d–g) Correlation between SRGN, THEMIS2, SGK1, FPR3, and infiltrating immune cells. ^∗^*P* < 0.05 and ^∗∗^*P* < 0.01. Correlation analysis was performed using Spearman's correlation analysis.

**Figure 5:** Experimental validation of SRGN function in the liver. (a) Oil Red O staining verified that FFA promoted lipid droplet formation. (b) Expression levels of SGRN, THMISE2, SGK1, FPR3, and lipid metabolism-related pathways in HepG2 after FFA induction. (c) Verification of SRGN transfection efficiency by qRT-PCR. (d) Western blot analysis revealed marked reductions in FASN and SREBP-1c protein expression levels in the cells after the silencing of SRGN while the protein expression levels of SIRT1 increased. (e) DEG levels in HepG2 cells were analyzed by fluorescence. (f) The silencing of SRGN reduced the formation of lipid droplet. ^∗^*P* < 0.05 and ^∗∗^*P* < 0.01.

**Table 1:** Data resource.

ID	Status	Organism	Tissue
GSE83452	Pre-BS (*n* = 16), post-BS (*n* = 16)	Homo sapiens	Liver biopsy
GSE106737	Pre-BS (*n* = 21), post-BS (*n* = 21)	Homo sapiens	Liver biopsy

**Table 2:** Primer sequences.

Gene	Sequences (5′-3′)
SRGN F	GGACTGACCTTTTTCCAAAGAC
SRGN R	GTCAAGAGACCTAAGGTTGTCA
THEMIS2 F	GGGTCTACTTCGAGGGCTCCATC
THEMIS2 R	TCTGGCTGGTCTTCGGGTTCTC
SGK1 F	CCCAACGACCTACGGCACTTTG
SGK1 R	CTTCCTTGACGCTGGCTGTGAC
FPR3 F	GCTGCCTCAACCCAATTCTCTACG
FPR3 R	GTGGTGTCTGTGTTGCTGGTCTG
SREBP-1 F	GCTGTTGGTGCTCGTCTCCTTG
SREBP-1 R	GCTTGCGATGCCTCCAGAAGTAC
SIRT1 F	AACAGGTTGCGGGAATCCAAAGG
SIRT1 R	CTCCTCGTACAGCTTCACAGTCAAC
FAS F	TCATCAAGGAATGCACACTCACCAG
FAS R	AAGAAGAAGACAAAGCCACCCCAAG
GAPDH F	CATGTTCCAATATGATTCCAC
GAPDH R	CCTGGAAGATGGTGATG

**Table 3:** Differentially expressed genes after bariatric surgery.

Differentially expressed genes	Gene names
Upregulated	TTN, PPARA, LINC00939, RPL19P12, DMRTA1, JAKMIP2, TPPP2, FOLH1, METTL7B, PKHD1, APOF, MOGAT1, MIR192, A2M, NECAB2, SLN, HNF1A-AS1, NEB, LOC100505918, XIRP2, STEAP1, CA14, SHBG, LOC730101, IGF1, CMYA5
Downregulated	JUN, MT1H, CXCL10, DUSP1, DDIT4, AVPR1A, MT1M, MIR21, SRGN, UPP2, NOCT, IGFBP1, ACSL4, ASCL1, SIK1, SDS, TP53INP1, MT1F, MT1A, FST, KLF6, CXCR4, MT1E, CXCL9, TMEM45B, C8orf4, APOA4, RGS1, S100A8, JUNB, JUND, NRG1, SAA1, RHOB, SGK1, LURAP1L, LAPTM5, MT1G, OSBPL11, S100A12, PDE11A, CXCL2, INSIG1, PRAMEF10, VTRNA1-1, FPR3, IP6K3, SYBU, MFSD2A, ZBTB16, TXNIPMT1L, FAT1, ARRDC4, LRRC31, LDLR, FGF21, KLF10, ATF3, TYROBP, FOS, BIRC3, THEMIS2, SQLE, PLIN2, PEG10, S100A9, THBS1SLC25A15, CCL4L2, TIMD4, ETNPPL, FGL2, CLGN, NAMPT, GDF15, VSIG4, NCAM2, FOSL2, PFN1P2, FADS1, SDC4, NNMT, CTSS

## Data Availability

All the data related to the research are included within this article. GSE83452 and GSE106737 can be found in the GEO database.
